The article "Machine Learning for Ischemic Heart Disease Diagnosis Aided by Evolutionary Computing" was retracted in 2023. Reasons: signs of a paper mill; compromised peer review; unreliable results or conclusions.

# Machine Learning for Ischemic Heart Disease Diagnosis Aided by Evolutionary Computing

**DOI:** 10.1155/2021/6718029

**Published:** 2021-11-17

**Authors:** Mohammad Alsaffar, Abdullah Alshammari, Gharbi Alshammari, Saud Aljaloud, Tariq S. Almurayziq, Fadam Muteb Abdoon, Solomon Abebaw

**Affiliations:** ^1^University of Ha'il, College of Computer Science and Engineering, Department of Computer Science and Information, Saudi Arabia; ^2^Analytical Chemistry, College of Sciences, Tikrit University, Iraq; ^3^Department of Statistics, Mizan-Tepi University, Ethiopia

## Abstract

Heart disease is the leading cause of death from chronic diseases in the developing countries. The difficulty of making an accurate and timely diagnosis is exacerbated by a lack of resources and professionals in some areas, which contributes to this reality. Medical professionals may benefit from technological advancements that aid in the accurate diagnosis of patients. In light of these findings, a hybrid diagnostic tool has been developed that combines several computational intelligence (machine learning) techniques capable of analyzing clinical histories and images of electrocardiogram signals and indicating whether or not the patient has ischemic heart disease with up to 97.01% accuracy. Working with medical experts and a database containing clinical data on approximately 1020 patients and their diagnoses was required for this project. Both were put to use. A picture database containing 92 images of electrocardiogram signals was also used in this project for the analysis of the Artificial Neural Network. After extensive research and testing by the medical community, which supported the project and provided positive feedback, a successful tool was developed. This demonstrated the tool's effectiveness.

## 1. Introduction

The relevance of the issue described here [1] is increased by the intricacy and importance of medical diagnosis, which can lead to disastrous outcomes if errors are made. Hussain et al. go on to say that because diagnosis is primarily an intuitive activity, it is impossible to say that every diagnosis is made without errors. Furthermore, there is a shortage of experts in various specialties in various areas, and no doctor, no matter how talented, is capable of attending to all specialties. These characteristics contribute to a favourable environment for the development and dissemination of intelligent tools that can help to decrease the complexity of diagnostic work, resulting in a number of benefits for society as a whole [2]. This work is to define the degree of correlation between each of the attributes/symptoms analyzed with the final diagnosis. Currently, the diagnostic process is carried out with little or without any support from intelligent tools, which is a totally subjective process, even when these professionals use more conclusive exams such as electrocardiogram signs, whose interpretation may vary from professional to professional. It should be noted that the Cardio Care work does not seek to replace the specialist medical professional but rather to serve as a support system for the decision-making process. There are currently many solutions designed to support the work of medical specialists [3], which proposes the realization of tele diagnosis and second opinion from a metropolitan computer network in Recife/PE, supported by two large local hospitals. In this proposal, hospitals are responsible for supporting others in Iraq with the accurate diagnosis of patients. Thus, the idea is to keep the specialist's attribution of weights but present a way to support this decision with the automatic calculation of the weights of the characteristics. The main objective of this work is to propose the development of a hybrid tool, where it is possible to record the experiences of medical specialists, especially those related to the studied domain (ischemic heart disease), later allowing the system to use this knowledge to solve future problems through application of artificial intelligence techniques (Case-Based Recognition, Genetic Algorithms, and Artificial Neural Networks).

The article "Machine Learning for Ischemic Heart Disease Diagnosis Aided by Evolutionary Computing" was retracted in 2023. Reasons: signs of a paper mill; compromised peer review; unreliable results or conclusions.

This research intends to test the following hypothesis: The best solution is determined by the AG, whose weights for the global similarity function (given by the weighted Euclidean distance) of the RBC and whose acuity will assist the medical specialist in the diagnosis of ischemic heart disease. It also tests the hypothesis that through the use of CI, it is possible to determine a higher rate of correct answers for the real diagnoses for this disease through the analysis of ECG signals, which will be analyzed by the tool itself.

## 2. Methodology

### 2.1. Data Collection and Analysis

For the preparation of this work, a database containing approximately 997 records was used, of which 592 had positive diagnoses for ischemic heart disease. We also used images extracted from the bunch of electrocardiogram signal images, acquired through the website of the European Union and European Society of Cardiology, which contains 92 freely distributed electrocardiogram image records, each being a result of 10 minutes of monitored signals duly noted by cardiologists. Finally, for the selection of the attributes to be considered as the most relevant and the primary definition of the relevance of each one, the work of Seitan, Venkatachalam and Hani (2009) [4] was carried out, from where the attributes were collected for the preparation of a questionnaire sent to several medical specialists for validation of the attributes and primary lifting of weights.

The article "Machine Learning for Ischemic Heart Disease Diagnosis Aided by Evolutionary Computing" was retracted in 2023. Reasons: signs of a paper mill; compromised peer review; unreliable results or conclusions.

### 2.2. Techniques, Features, and Settings

This work used the following techniques related to computational intelligence: Genetic Algorithms, Case-Based Reasoning, Computer Graphics, and Artificial Neural Networks.

The proposed solution offers the user not only support for the decision-making process but also operational support for the activities of a clinic or doctor's office. The environment used for the development of this tool was as follows:

- Software:

- Operating System Windows 10
- Development Platform, Visual C# Express
- C# Programming Language

(b) Hardware:

- Notebook
- Intel Core i3 Processor—Second Generation
- 8 GB RAM memory

All technology used to develop the tool in question can be acquired at a relatively low cost by organizations that promote public and/or private collective health.

### 2.3. Algorithms

The proposed tool basically applies the following key algorithms for its correct functioning: Genetic Algorithms (for case-based reasoning module), computer graphics algorithms (based on the OTSU algorithm), and Artificial Neural Networks algorithm—MPL—back rogation, used from the import of the FANN library (Fast Artificial Neural Network).

### 2.4. Computer Graphics/Artificial Neural Networks (ANN)

Seeking to offer a second diagnosis or even the possibility of carrying out diagnostic indications based on images of electrocardiogram signals, the ANN module was implemented. However, for this module to work correctly, it was necessary to convert the images (scanned or retrieved directly in digital form) into binary matrices, thus allowing the generation of the necessary inputs for the ANN. In order for the solution to be able to perform a diagnostic indication by image analysis, the user must first perform system training by retrieving the image which, after being submitted to the appropriate algorithms (which can be seen in the appendices) will generate the entries necessary for ANN training.

The algorithm used in this work receives as input the file containing information about the images for training (input bits and output bit). The output bits are represented by 0 (absence of the disease) and 1 (presence of the disease), the ANN being able to return any value between these ranges indicating the degree of indication. Once the training is done, the function returns the network configuration file for future use.

## 3. Results and Discussion

Since the solution presented is a hybrid tool that combines different technologies and modules, each presenting separate results (which can be grouped and compared by the user's option to generate a single result), in the tests and simulations, it was addressed the concept of proof and reproof. The same test was then applied in the RBC and ANN module, with the results being divided by module, thus seeking better readability and understanding for the reader. Soon, the results were organized like this.

The article "Machine Learning for Ischemic Heart Disease Diagnosis Aided by Evolutionary Computing" was retracted in 2023. Reasons: signs of a paper mill; compromised peer review; unreliable results or conclusions.

### 3.1. ANN Results

After carrying out the training in which the aforementioned specifications were used, it was possible to observe the evolution of ANN as new cases were submitted to the test. In the simulations, an average error curve similar to that shown in Figure 1 can be observed, which corresponds to the result of the ANN training process, for diagnosis of ischemic heart disease based on clinical data, that is, without performing any analysis on the images of the ECG signals.

It can be seen from the figure that, as the training progresses, there is also a reduction in the average error rate, with the system reaching a point of minimum convergence between the 4000 and 4500 times; thus, it is not necessary to continue with the training.

When undergoing training for image analysis of electrocardiogram signals, ANN presented the following mean error curve figure, see Figure 2.

In training for pattern recognition and diagnostic indication based on the analysis of electrocardiogram signals, the network presents stagnation in the evolution of the correctness rate even before the 2500th epoch, and then, its training may be ended. Then, overlaying the evolution of ANN for the two trainings, Figure 3 is obtained.

It is possible then to note that, despite being tenuous, there is a superiority in the hit rates of trained ANN for clinical data over ANN trained for image analysis of EGC signals, which can on the one hand be explained, for example, due to need to process and convert images that can lead to some loss of information.

The information obtained during the training and simulation process of the ANN module provided support for the definition of the following table of results, see Table 1. This confirms, as can be seen in the table above, the capacity reached by ANN to diagnose the disease studied from the analysis of clinical data from the patient's history and/or through the simple analysis of ECG signs.

### 3.2. RBC (Case-Based Reasoning) Results (AG)

As performed in the ANN module, the RBC by AG module was subjected to various testing and simulation procedures. The data and configurations used for the processes were discussed previously, as well as the methods applied. After testing and simulation performing the procedures, the algorithm returned the following evolution to Figure 4.

The article "Machine Learning for Ischemic Heart Disease Diagnosis Aided by Evolutionary Computing" was retracted in 2023. Reasons: signs of a paper mill; compromised peer review; unreliable results or conclusions.

The chart above shows the evolution of solutions for each generation. The darker line represents the best fitness of each generation (Figure 4) while the lighter lines represent the average fitness of the generation. It can be seen from the figure that the peak of the algorithm occurs in the 12th generation, after which it presents variations with a negative trend, as can be seen in Figure 5 of convergence analysis.

The figure above shows the negative trend of future results; however, it cannot be said with complete certainty that, from the 20th generation onwards, solutions with better fitness will not emerge. However, the negative trend indicated by the convergence curve indicates an opposite situation, which justifies the interruption of the tests.

At the end of the tests, the algorithm reached hit peaks of up to 99%; however, the accepted value for validation of the results was the average hit rate, which reached values of up to 97.01%. After training, all values (weights) generated by each of the individuals in each of the generations were recorded in a database for future analysis; the 9 best individuals/solutions were also separated for comparison with the data reported by the group of medical experts, thus resulting in Table 2.

Table 2, as already described, presents values of the 9 best individuals found by the solution. These individuals were selected so that the means of each attribute could be calculated with the same number of samples obtained through the weights assigned by the experts. Table 2 also presents the comparison between the results.

Once the points of divergence are identified, it is possible to carry out a more accurate survey of the attributes that deserve more attention from specialists, even allowing for a discussion with them to improve the tool and their work.

### 3.3. Validation

After analyzing the results of the weights applied to each analyzed attribute, the tool in question, here called AP04, was compared with other applications with similar purposes, in addition to the traditional method itself. The comparisons that sought to prove the equivalence of quality of the application presented in relation to other methods available in the literature took into account three tools proposed by international journals [5], presenting in their work a hybrid tool based on logic fuzzy with rates of up to 93.27% hits (AP01), also developing a hybrid tool based on fuzzy logic, obtained hit rates in the order of 91.58% (AP02) and proposed an online application capable of reaching up to 86.1% of acuity (AP03). The percentage of correct answers of traditional methods (TRAD) was calculated based on the database used for training the application proposed here, since this database contained not only the real diagnoses but also those indicated by the medical professional. In Table 3, it is possible to observe the results of the comparative process, where statistical methods of calculation of variance were applied [6], thus preparing for the application of other methods that classify the tool in relation to the others with to which it has been compared.

The article "Machine Learning for Ischemic Heart Disease Diagnosis Aided by Evolutionary Computing" was retracted in 2023. Reasons: signs of a paper mill; compromised peer review; unreliable results or conclusions.

It is noted in Table 3 that, from each tool/method, 10 samples were taken at random, and the comparative methods are presented, and the methods applied for analysis of variance; the summary presented in Table 4 was obtained.

Subsequently, the data was submitted to analysis of variance (ANOVA) seeking to confirm or reject the hypothesis of equality between the means, resulting in the tables shown in Table 4.

In addition the overall hit rates of each one of them to having been tested for its overall ability to correctly indicate positive or negative diagnoses for the disease studied. Once the system was calibrated and the weights of each of the attributes distributed as indicated in the previous tables, it was subjected to new evaluations, now seeking to measure its rate of specificity, sensitivity, prevalence, and accuracy, whose importance was once highlighted by Flores [7], when it comes to clinical and laboratory analyses, tools, methods, or other operations that mention the medical or clinical diagnosis that should always demonstrate the results of these tests.

For the analysis of these tests, the system was submitted to new simulations; this time being randomly selected and using 500 records taken from the database used for training the algorithm. Such records were selected to compose a simulation base, which is responsible for making the inputs to the system simulating its use, recording all the results necessary to carry out the aforementioned tests, and generating, after due analysis, the results presented in Table 5.

It is also the process used to make sparkling wines (not named “Champagne”) in different French areas, as well as Cava in Spain, Espumante in Portugal, and Franciacorta in Italy. The process is known as the method champ noise, but Champagne producers have successfully pushed the European Union to limit the term's usage within the EU to Champagne wines exclusively.

Still following the concepts presented by Flores [8–27], it can be said that the tests performed allow to define the real capacity presented by the tool to present positive results, for patients who really have ischemic heart disease (sensitivity); specificity refers to measuring the tool's ability to indicate and diagnose a true negative, that is, to indicate that an individual is healthy when he/she really does not have ischemic heart disease; the number of tested cases within all selected for the simulations is given by the prevalence; finally, the veracity of the test, that is, how much the test approaches or departs from the “truth,” is given by its accuracy.

The article "Machine Learning for Ischemic Heart Disease Diagnosis Aided by Evolutionary Computing" was retracted in 2023. Reasons: signs of a paper mill; compromised peer review; unreliable results or conclusions.

All results obtained by the tool, with regard to the tests mentioned above, were also confronted with results obtained through different methods and tools also intended for this purpose (Almeida, [28]), which are cited as follows: Fisher's Linear Analysis (Fisher), Decision Trees (AD), Logistic Regression (RL), and Artificial Neural Networks (ANN), in addition to the method proposed here, Genetic Algorithms with Case-Based Recognition (AG + RBC).

It can be seen the comparison that the method proposed here presents sensitivity rates very close to those presented by Fisher's linear model, which, of the methods in question, presented the best rate. As for the specificity, the rates were very close to the models of Decision Trees, Logistic Regression, and Artificial Neural Networks, which were the methods with the best results, thus demonstrating that the tool proposed here presents results that fit into the group of solutions (found in the bibliography accessed) which present the most expressive results.

## 4. Conclusions

The main objective of the work is to present a specific decision support tool for the diagnosis of ischemic heart disease, with possibilities for adaptation and learning so that it can be used in the diagnosis of other diseases. This tool is presented as an option to existing solutions, in which a hybrid proposal is applied, combining characteristics of evolutionary computing (Genetic Algorithms) and machine learning (Case-Based Reasoning and Artificial Neural Networks). Thus, in addition to predicting diagnoses through the analysis of clinical data, the system also became capable of analyzing images of electrocardiogram signals, thus offering medical professionals more information to support their decision.

Dividing the analysis of the proposal into modules, the one in which evolutionary computing was applied and the one in which ANN was applied, it can be concluded that the results presented in the performed experiments (considering only the evolutionary computing module) show that the proposed application presents hit rates significantly higher than the other applications with which it was compared, proving to be even more efficient when compared to traditional diagnostic methods. The ANN module has lower rates and may fit the same hit rates of traditional methods; however, it should be considered that the ANN module has lower results when only ECG signal image analysis is used as inputs, excluding if the other findings of the clinical analyses, leading to the belief that the tool has great capacity for classification and diagnostic prediction, even with a reduced amount of information, it being sufficient for this information to have a high degree of relevance, which is also computed by the tool. Given the results of the statistical analyses carried out to prove the good results presented by the proposed application, one can see the great advantages obtained through small adaptations made to the algorithms and the selection of a similarity function suitable for the problem in question, leading the application to results expressive in indicating the possibility of the presence of obstructive coronary disease in the cases analyzed, as well as good rates of specificity and sensitivity. Thus, based on the results, the tool proposed here fits into the levels of quality and ability to get it right observed in the main tools with the same purpose observed in the literature.

The article "Machine Learning for Ischemic Heart Disease Diagnosis Aided by Evolutionary Computing" was retracted in 2023. Reasons: signs of a paper mill; compromised peer review; unreliable results or conclusions.

## Figures and Tables

**Figure 1:** Average training error—clinical data.

**Figure 2:** Average training error—ECG signals.

**Figure 3:** Average training error—ANN overlay—clinical data × ANN ECG images.

**Figure 4:** Algorithm evolution—maximum and average hits.

**Figure 5:** Convergence analysis.

**Table 1:** Configuration and results of the ANN's learning process (source: the author).

Number of neurons	Epochs	Apprenticeship	Activation function	Training %	Test %	Source data
5	3700	0.3	Sigmoid	81.4	81.5	Clinical
5	3700	0.3	Sigmoid	91.3	80.9	Image
10	2709	0.7	Sigmoid	90.9	80.9	Clinical
10	2342	0.7	Sigmoid	79.4	78.9	Image
15	1876	0.9	Sigmoid	87.0	87.0	Clinical
15	1765	0.9	Sigmoid	85.1	84.9	Image
20	3200	0.3	Sigmoid	76.7	75.0	Clinical
20	3100	0.3	Sigmoid	89.0	89.0	Image
25	2903	0.7	Sigmoid	83.3	82.3	Clinical
25	2876	0.7	Sigmoid	82.2	82.2	Image

**Table 2:** Weights assigned by the AG and comparison—averages of the weights assigned by the experts and the AG.

	Weights assigned by the AG										Comparison—averages of the weights assigned by the experts and the AG			
Attribute	1	2	3	4	5	6	7	8	9	Average	Average specialists	Average AG	Variation	
Age	0.8	0.8	0.8	0.8	0.8	0.27	0.8	0.8	0.8	0.74		0.43	0.74	0.31
Sex	0.2	0.2	0.2	0.2	0.2	0.47	0.2	0.47	0.2	0.26	0.45	0.26	0.19	
Systolic pressure	0.53	0.53	0.6	0.53	0.53	0.53	0.53	0.53	0.53	0.53	0.33	0.53	0.2	
Diastolic pressure	0.47	0.47	0.47	0.47	0.47	0.47	0.47	0.47	0.47	0.47	0.43	0.47	0.04	
Heart rate	0.8	0.8	0.8	0.8	0.8	0.53	0.8	0.8	0.8	0.47	0.53	0.47	0.06	
Pain intensity	0.47	0.47	0.47	0.47	0.47	0.47	0.47	0.47	0.47	0.54	0.37	0.54	0.17	
Start time of last pain episode	0.53	0.53	0.8	0.8	0.53	0.67	0.53	0	0.53	0.47	0.52	0.47	0.05	
Symptom onset time	0.47	0.47	0.47	0.47	0.47	0.47	0.47	0.47	0.47	0.53	0.37	0.53	0.17	
Background	0.53	0.53	0.53	0.53	0.53	0.53	0.53	0.6	0.53	0.47	0.85	0.47	0.38	
Pain characteristic	0.47	0.47	0.47	0.47	0.47	0.47	0.47	0.47	0.47	0.57	0.63	0.57	0.06	
Changes in the electrocardiogram	0.53	0.67	0.53	0.53	0.8	0.53	0.53	0.53	0.53	0.47	0.61	0.47	0.14	
Pain site	0.47	0.47	0.47	0.47	0.47	0.47	0.47	0.47	0.47	0.56	0.76	0.56	0.2	
Other symptoms	0.53	0.53	0.53	0.53	0.53	0.8	0.53	0.53	0.53	0.46	0.8	0.46	0.34	
Auscultation signals	0.47	0.47	0.4	0.47	0.47	0.47	0.47	0.47	0.47	0.46	0.52	0.46	0.06	
Observed signs	0.6	0.53	0.53	0.53	0.53	0.53	0.53	0.8	0.53	0.56	0.57	0.56	0.01	
Risk factors	0.47	0.47	0.4	1	0.47	0.47	0.47	0.47	0.33	0.5	0.56	0.5	0.06	
Pulse signals	0.53	0.53	0.53	0.53	0.53	0.53	0.53	0.67	0.53	0.53	0,31	0,53	0,22	

The article "Machine Learning for Ischemic Heart Disease Diagnosis Aided by Evolutionary Computing" was retracted in 2023. Reasons: signs of a paper mill; compromised peer review; unreliable results or conclusions.

**Table 3:** Comparison between tools and traditional method—variance.

	Group				
	AP01	AP02	AP03	AP04	TRAD
1	89.10	88.73	85.71	94.08	88.05
2	90.53	90.16	87.08	95.59	89.46
3	89.73	89.36	86.31	94.75	88.67
4	92.02	91.64	88.52	97.16	90.94
5	91.98	91.60	88.48	97.12	90.90
6	93.23	92.85	89.68	98.44	92.13
7	92.12	91.74	88.61	97.27	91.03
8	93.27	92.89	89.72	98.48	92.17
9	93.01	92.63	89.47	98.21	91.91
10	93.26	92.88	89.71	98.47	92.16
Summary					
Score	10.00	10.00	10.00	10.00	10.00
Sum	918.25	914.49	883.30	969.58	907.43
Average	91.83	91.45	88.33	96.96	90.74
Variance	2.3061	1.0336	1.1409	1.0469	0.4298

**Table 4:** ANOVA and Tukey test.

ANOVA							Tukey		
	SQ	gl	MQ	F	*p* value	F-critical	Group	Average	Class
Variance source	891.93	4	222.98	187.165	2.01*E*-27	2.5787	AP04	96.9	A
Between groups	63.511	46	1.1914				AP01	91.8	B
							AP02	90.5	B
Total	945.548	49					TRAD	46.4	C
							AP03	85.02	C

**Table 5:** Comparison between tools and traditional method—variance.

Legend	Values	Observations
Total simulations	500	
Positive indications	289	
True positive (VP)	13	
False positives (FP)	177	
Negative indications	162	
True negatives (VN)	15	
False negative (FN) sensitivity	95.05%	VP/(VP + FN)
Specificity	92.57%	VN/(FP + VN)
Prevalence	63.46	(VP + FN)/(VP + FN + VN + FP)
Accuracy	96.86	(VP + VN)/(VP + FN + VN + FP)

## Data Availability

The data utilized to back up the study's conclusions are given in the article.
